# Enhancement of oxidation resistance via a self-healing boron carbide coating on diamond particles

This article has been retracted.

**DOI:** 10.1038/srep20198

**Published:** 2016-02-02

**Authors:** Youhong Sun, Qingnan Meng, Ming Qian, Baochang Liu, Ke Gao, Yinlong Ma, Mao Wen, Weitao Zheng

**Affiliations:** 1 College of Construction Engineering, Jilin University, Changchun 130026, People’s Republic of China; 2 Key Lab of Drilling and Exploitation Technology in Complex Conditions, Ministry of Land and Resources, Changchun, 130061, People’s Republic of China; 3 State Key Laboratory of Superhard Materials, Jilin University, Changchun 130012, People’s Republic of China; 4 Department of Materials Science, Jilin University, Changchun 130012, People’s Republic of China

## Abstract

A boron carbide coating was applied to diamond particles by heating the particles in a powder mixture consisting of H_3_BO_3_, B and Mg. The composition, bond state and coverage fraction of the boron carbide coating on the diamond particles were investigated. The boron carbide coating prefers to grow on the diamond (100) surface than on the diamond (111) surface. A stoichiometric B_4_C coating completely covered the diamond particle after maintaining the raw mixture at 1200 °C for 2 h. The contribution of the boron carbide coating to the oxidation resistance enhancement of the diamond particles was investigated. During annealing of the coated diamond in air, the priory formed B_2_O_3_, which exhibits a self-healing property, as an oxygen barrier layer, which protected the diamond from oxidation. The formation temperature of B_2_O_3_ is dependent on the amorphous boron carbide content. The coating on the diamond provided effective protection of the diamond against oxidation by heating in air at 1000 °C for 1 h. Furthermore, the presence of the boron carbide coating also contributed to the maintenance of the static compressive strength during the annealing of diamond in air.

Diamond has the highest hardness and excellent thermal conductivity, making it useful for reinforced composite materials, such as diamond compacts, which are potential candidates for use in a variety of applications, such as drill bits, saw blade segments, grinding wheels, cutting and polishing tools, and heat sinks for electronic devices^1^,^2^,^3^,^4^,^5^. The manufacturing process of diamond tools requires a high temperature. However, the oxidation of diamond occurs at approximately 700 °C in air, which leads to catastrophic loss of its mechanical properties and limits its wide applications under oxidizing conditions. Therefore, high temperature oxidation protection of diamond is very important for practical applications of diamond tools.

Boron oxide (B_2_O_3_) has many advantageous properties that make it useful for oxidation protection applications. B_2_O_3_ possesses low oxygen permeability, higher fluidity and good wettability on carbon materials below 1000 °C, which results in self-healing coatings on carbon materials^6^,^7^,^8^,^9^,^10^,^11^. However, when exposed to ambient moisture, hydrolysis of B_2_O_3_ causes the glass to swell and crumble, which can result in coating spallation at room temperature due to glass swelling or spallation during heating due to moisture release^12^. Hydrated borate (i.e., Na_2_B_4_O_7_•10H_2_O) is a common substitute. However, the usefulness of borate glasses is also limited because hydrated borates are highly volatile. Therefore, glass depletion may occur at relatively low temperatures in moist environments^13^. Doping boron into diamond is an effective route for improving the oxidation resistance of diamond. Many studies have demonstrated that the oxidation resistance of boron-doped diamond increases as the boron content increases, and different mechanisms for boron inhibition have been proposed^14^,^15^,^16^. The main disadvantage of boron-doped diamond is the degradation of the crystallinity. The Raman spectra in ref. 14 indicate that an increase in the boron content results in a broader diamond peak as well as other impurity peaks (amorphous structures). Zhang *et al.*^17^ have also reported that the percentage of high-quality crystals of high-pressure high-temperature (HPHT) diamond continually decreased as the boron content increased.

Boron carbide (B_4_C) coatings are of interest due to their potential use for improving the oxidation resistance of diamond. The oxidation of B_4_C occurs at approximately 700 °C and forms a B_2_O_3_ oxygen barrier^18^. In addition, B_4_C is a refractory hard material that is insoluble in water and chemically inert below 700 °C 19. These reasons suggest that a boron carbide coating has the potential to improve diamond oxidation resistance. However, high quality B_4_C requires a high synthesis temperature and long holding time^19^,^20^,^21^ because the process is highly endothermic and requires 16,800 kJ/mol B_4_C^22^. Recently, Ras *et al.*^23^ have successfully synthesized a B_4_C coating on diamond particles using a mixture of B and H_3_BO_3_ as the boron sources. The nucleation of B_4_C was obtained after 2 hours of holding at 1050 °C, and complete coverage of the diamond particles with B_4_C was achieved after 6 hours of holding at 1150 °C. However, the product quality of the coating (e.g., composition) has yet to be report. Hu and Kong^3^ have also synthesized a B_4_C coating on diamond particles using the same method that was reported in ref. 23 at 850 °C. However, a large amount of graphite was obtained based on the X-ray photoelectron spectroscopy (XPS) analysis. In addition, the influence of the synthesis temperature on the nucleation and growth of the B_4_C coating on different surfaces of a single crystal diamond has not been previously studied. Moreover, the influence of the boron carbide coating on the enhancement of the oxidation resistance of diamond particles has not been previously investigated.

In this study, the ability of a boron carbide coating to protect diamond and improve its oxidation resistance has been studied. During annealing of the coated diamond in air, a B_2_O_3_ oxygen barrier layer formed prior to the oxidation of diamond. In addition, fluidic B_2_O_3_ results in a self-healing property that can repair defects (e.g., hole and blank). Therefore, the coating can impede corrosion of diamond from the oxygen in air at a high temperature.

## Results

Figure 1 shows the X-ray diffraction (XRD) patterns for the uncoated (D0) and coated diamond particles (D1-3). As shown in Fig. 1, the peak located at 43.92 degrees was observed in all the spectra, which corresponds to diamond (JCPDF#06-0675). To clearly observe the other peaks for the coating on the diamond particle, a high-intensity peak for the single crystal diamond substrate was partially truncated. In addition, three peaks located at 23.33°, 34.73° and 37.56° were observed for coatings synthesized at 800 (D1) and 1000 °C (D2), and three more low-intensity peaks located at 21.88°, 31.76° and 49.86° were observed for the coating synthesized at 1200 °C (D3). In comparison to the standard PDF cards shown in Fig. 1, these diffraction peaks can be assigned to the B_4_C, B_13_C_2_ or B_10_C structure. The following XPS and Raman results suggest that the phase structure of the coating is B_4_C. In addition, as shown in Fig. 1, a lower synthesis temperature resulted in broadening of the diffraction peaks for the boron carbide coatings. The grain sizes of the boron carbide coating calculated from Williamson-Hall plot increased from 36 to 64 nm as the synthesis temperature increased from 800 to 1200 °C.

The chemical bonding and composition of the boron carbide coatings on the (100) surface of diamond particles were studied by XPS (Fig. 2). The composition and B:C atomic ratio are listed in Table 1. The results indicate that the B:C atomic ratio for the boron carbide coating on the diamond (100) surface increased from 3:1 to 4:1 as the synthesis temperature increased from 800 to 1200 °C, suggesting that the crystal structure determined by XRD (Fig. 1) is the B_4_C phase. The XPS C1s spectra for the boron carbide coatings on the (100) surface of the diamond particles synthesized at different temperatures are shown in Fig. 2a, and two peaks can be identified. The peak located at 285.2 eV was assigned to C-C bonds^24^, and the peak located at 282.4 eV was due to C-B bonds^25^. The contribution from the C-C bonds decreased as the synthesis temperature increased and nearly disappeared when the synthesis temperature reached 1200 °C. Fig. 2b shows the XPS B1s spectra for the boron carbide coatings on the (100) surface of the diamond particles synthesized at different temperatures. The main peak in all the B1s spectra is located at 187.5 eV, which corresponds to typical B-C bonds^15^,^26^. Moreover, the spectrum for the boron carbide coating on the diamond particles synthesized at 800 °C (D1) exhibits a shoulder at 188.8 eV, which was due to amorphous boron carbide (denoted B-C*)^15^,^26^,^27^. The fraction of B-C* bonds in the B1s spectrum significantly decreased as the synthesis temperature of the boron carbide coating decreased and completely disappeared when the synthesis temperature reached 1200 °C. The content of amorphous boron carbide in the coatings on the diamond particles synthesized at different temperatures calculated from the XPS analysis is also listed in Table 1. The content of amorphous boron carbide is strongly dependent on the synthesis temperature.

Raman analysis was performed using a confocal system. The Raman laser was forced on the (100) surface of the diamond particles to characterize the binding states of the boron carbide coating. Figure 3 shows the Raman spectra for all the samples in a range between 200 and 2000 cm^−1^. A high-intensity peak located at 1333 cm^−1^, which was observed in all the spectra, corresponded to diamond^28^. In agreement with the literature data, a series of bands extending from 200 to 1200 cm^−1^ were assigned to vibrations of the principal structural elements, icosahedra and three-atom linear chains in the B_4_C crystal^29^,^30^,^31^,^32^,^33^. In addition, the intensity of the peaks located at 269 and 325 cm^−1^ decreased as the synthesis temperature increased and completely disappeared when the synthesis temperature reached 1200 °C. These peaks are related to chain-icosahedral linkages of amorphous boron carbide^33^, which is in good agreement with the XPS analysis. Furthermore, the G peak located at 1550 cm^−1^ and D peak located at 1350 cm^−1^ 24 were not observed in the coating synthesized at 800 °C (D1), which indicates that graphitic carbon does not exist in the boron carbide coating on the diamond particles.

Figure 4 shows the scanning electron microscopy (SEM) images for the uncoated (D0, Fig. 4a) and coated diamond particles (D1-3, Fig. 4b–d). The coating coverage is dependent on the synthesis temperature. At 800 °C (D1), the diamond (100) surfaces (square surfaces^34^,^35^,^36^) are completely covered by the coating, as shown in Fig. 4b. However, only the nucleation of the coating on diamond (111) surfaces (triangle or hexagon surfaces^34^,^35^,^36^) occurred at this synthesis temperature. As the synthesis temperature increased, the coating starts to grow on the diamond (111) surface. Complete coverage of the diamond particles was achieved when the synthesis temperature reached 1200 °C (see Fig. 4d, sample D3). The typical SEM cross-section image for the boron carbide coating on different surfaces of diamond synthesized at 1200 °C (D3) are shown in Fig. 5. As the synthesis temperature increased from 800 °C (D1) to 1200 °C (D3), the thickness of the coating on the (100) surface increased from 1 to 3 μm. In addition, the thickness of the coating on the (111) surface for D3 was 2 μm.

All the samples were annealed at 1000 °C in an air atmosphere at a heating rate of 5 °C/min to characterize the oxidation resistance. The XRD patterns for the uncoated (A0) and boron carbide coated (A1-3) diamond particles after annealing are shown in Fig. 6. The diffraction peaks located at 14.56, 27.77 and 30.59° were assigned to the B_2_O_3_ structure, and the high-intensity peak corresponding to the single crystal diamond substrate (i.e., approximately 43.92°) was partially truncated. In addition, the grain size calculated using the Williamson-Hall plot in Fig. 6 was 14, 22 and 34 nm for the A1, A2 and A3 samples, respectively. The XPS B1s and O1s spectra for the coatings on the (100) surface of the diamond particles after annealing in an air atmosphere are shown in Fig. 7. In this case, only B-O bonds (193.6 eV^26^) and O-B bonds (533.6 eV^37^) were observed. The compositions of the coatings after annealing are also listed in Table 2. The B:O atomic ratio in all the coatings is close to 2:3, which is in good agreement with the XRD results (Fig. 6). In addition, it is important to note that the B-C* peak located at 188.8 eV, as shown in Fig. 2b but not in Fig. 7a. This result indicates that amorphous boron carbide was also oxidized during the annealing process.

To further investigate the binding states of the coatings on the diamond particles after annealing in air, Raman spectroscopy was employed (see Fig. 8). In addition to the diamond peak at 1333 cm^−1^, the Raman spectra for all the coatings after annealing in air contain two sharp peaks at 1360 and 1400 cm^−1^, which are assigned to B-O bonds^38^. In comparison to the Raman results prior to annealing in air (Fig. 3), the peaks for the B_4_C crystal located in a range from 400 to 1200 cm^−1^ disappeared, which suggests that B_4_C was oxidized during the annealing process. This result confirms the XRD (Fig. 6) and XPS (Fig. 7) results. Moreover, D and G peaks (1350 and 1550 cm^−1^) rather than amorphous boron carbide peaks (269 and 325 cm^−1^) were observed in the Raman spectra for samples A1 and A2. The use of a higher synthesis temperature to prepare the boron carbide coating results in a lower contribution from the D and G peaks after annealing. The D and G peaks were not observed in the Raman spectrum for sample A3, which indicates that amorphous boron carbide was also oxidized during the annealing process, and a larger amount of amorphous boron carbide contributed to the formation of amorphous carbon. Furthermore, the formation of amorphous carbon restricts grain growth of the B_2_O_3_ crystal during annealing, resulting in a refined B_2_O_3_ crystal grains in A1, as shown in Fig. 6.

Detailed thermal analyses of all the samples were performed using thermal gravimetric analysis (TGA). The temperature for the TGA was programmed to increase from room temperature (20 °C) to 1000 °C at a rate of 5 °C/min, and then, the temperature was maintained at 1000 °C for 4 h. The results of the TGA measurement for the uncoated (D0) and boron carbide coated diamond (D1-3) particles are shown in Fig. 9. For the uncoated diamond particles (D0), the TGA curve exhibits an abrupt decrease from 100.0 to 45.5% when the testing temperature increased from approximately 720 to 1000 °C, indicating that the diamond was not oxidized until 720 °C. All the diamond particles with boron carbide coating (D1-3) exhibited a weight gain in a temperature range from 300 to 1000 °C. Along with the XRD (Fig. 6), XPS (Fig. 7) and Raman (Fig. 8) results, the weight gain was due to the formation of B_2_O_3_. During holding at 1000 °C, the coated diamonds exhibited a slow decrease in their weight due to evaporation of B_2_O_3_. When the protective B_2_O_3_ completely evaporates, the samples exhibited a significant decrease in weight due to the oxidation of diamond. As shown in Fig. 9b, the boron carbide coating on the diamond is beneficial for delaying the oxidation of diamond. In this study, the coating on the diamond (sample D3) can provide effective protection against oxidation by heating in air at 1000 °C for 1 h. In comparison to the uncoated diamond particles, the initial time prior to the oxidation of diamond was delayed by 2 h.

Figure 10 shows the SEM images for the uncoated (A0, Fig. 10a) diamond particles and boron carbide coated diamond particles (A1-3, Fig. 10b–d) after annealing using a heating rate of 5 °C min^–1^ in an air atmosphere. As shown in Fig. 10a, the edges and corners of the uncoated single crystal diamond particle (A0) disappeared after annealing. In contrast, the diamond particles with the boron carbide coating (A1-3, Fig. 10b–d) possess a complete coverage of edges and corners after annealing. In addition, a slight oxygen corrosion pit was observed on the diamond (111) surface of sample A1, leading to a slight weight loss at high temperature (see Fig. 9). For samples A2 and A3, the surface of the diamond particles was completely covered by the B_2_O_3_ coating, and no oxygen corrosion pit was observed.

The static compressive strengths of one diamond particle from each of the samples are shown in Fig. 11. For diamonds with boron carbide coatings that were synthesized in a vacuum (D1-3), the static compressive strengths were nearly constant at approximately 175 N, which similar to the result for the uncoated diamond particles (D0). After annealing in air, the static compressive strengths of the uncoated diamond particles (A0) decreased to 86 N. In contrast, in comparison to the results for D2 and D3, the corresponding samples after annealing in air (A2 and A3) maintain the same level of static compressive strength.

## Discussion

In combination with the XRD (Fig. 1), XPS (Fig. 2) and Raman (Fig. 3) results, boron carbide coated the diamond particles due to heating the diamond with a mixture of B, boric acid (H_3_BO_3_), and magnesium (Mg). After holding the raw mix at 1200 °C for 2 hours (Sample D3), the coating on the diamond exhibited a stoichiometric B_4_C crystal structure without any impurities or amorphous structures. The overall reaction can be expressed as^39^,^40^,^41^



This reaction proceeds in the following three steps.







In this case, B_2_O_3_ is reduced by Mg (eq. 3), which makes the overall reaction (eq. 1) exothermic (ΔH = 1812 kJ/mol) in nature^19^. In addition, Mg also provided active sites for the nucleation of B_4_C, resulting in a reduction of the synthesis temperature of B_4_C^41^. Furthermore, the crystallization and growth rates of B_4_C were dependent on the synthesis temperature. The thickness of the coating on the (100) surface increased from 1 to 3 μm as the synthesis temperature increased from 800 to 1200 °C. In addition, the B_4_C grain size increased as the synthesis temperature increased. Furthermore, the amorphous structure content decreased. For the boron carbide coating synthesized at a lower temperature (800 °C, sample D1), a large amorphous content (29%) was observed based on the XPS (Fig. 2, Table 1) and Raman (Fig. 3) results. In ref. 39, an amorphous content of approximately 30% was also observed in the boron carbide powders synthesized at 700 °C with Mg and K_2_SO_4_ as catalysts. In ref. 42, a stoichiometric B_4_C crystal powder was obtained after holding at 800 °C according to the reaction described in equation 1. However, a long holding time (20 hours) was required.

The boron carbide coating on the diamond particles improved the resistance to oxygen corrosion by forming B_2_O_3_ as an oxygen barrier layer. Interestingly, the initial temperature of the weight gain for the diamond particles with the boron carbide coating synthesized at 800, 1000 and 1200 °C was 350, 500 and 700 °C, respectively (see Fig. 12), which are lower than the oxidation temperature of diamond (720 °C). In combination with the XPS (Fig. 2, Table 1) and Raman (Fig. 3) analyses, the initial temperature of the weight gain was dependent on the amorphous content in the boron carbide coating on the diamond particles, as shown in Fig. 12. A larger amount of the amorphous boron carbide structure shifts the initial temperature of the weight gain to a lower value because the amorphous boron carbide can be oxidized in air at a lower temperature^15^ The dependence of the B_2_O_3_ formation temperature on the amorphous boron carbide content suggests that the boron carbide coating with a higher amorphous content is a potential antioxidant material for the sample with a low oxidation temperature. In this study, all the boron carbide coatings are oxidized prior to the oxidation of diamond, which implies that the boron carbide coating can protect the diamond against oxidation due to previous formation of a B_2_O_3_ coating.

Based on the SEM analysis, the cover state of the coating on diamond is different for the same sample before and after annealing in air due to the self-healing of B_2_O_3_. Because the melting point of B_2_O_3_ (~450 °C) is much lower than the oxidation temperature of diamond (720 °C), indicating that the B_2_O_3_ formed during annealing exhibits fluidity. During annealing, the fluidity of B_2_O_3_ is beneficial for self-healing and densification of the protective coating on the diamond surface prior to oxidation, which improves the oxidation resistance of the diamond particles. Therefore, the slight oxygen corrosion observed on sample A1 (Fig. 10b) was only due to the crystal nucleus of boron carbide existing on the corresponding diamond (111) surface prior to annealing in air (Fig. 4b, D2). This coating contributed to the topical protection of the diamond (111) surface from being oxidized. However, a B_2_O_3_ coating that completely covers the diamond (111) surface during annealing is difficult to achieve. Furthermore, sample A2 was completely covered by the B_2_O_3_ coating (see Fig. 10c) even though the diamond (111) surface was only partially covered by the boron carbide coating for the corresponding sample prior to annealing (Fig. 4c). The oxidation of boron carbide leads to a 250% increase in volume^18^.

The static compressive strength of the diamond particle is dependent on the oxidation resistance of the diamond particles. The surface of the uncoated diamond after annealing exhibited severe corrosion by oxygen, and the corrosion pit contributed to the extension of the crack under compression. The TGA results and SEM images suggest that the coating on the diamond particles protect the diamond against oxidation, resulting in maintenance of the static compressive strength. As shown in Fig. 11, the static compressive strengths for A2 and A3 are the same as those for the corresponding samples prior to annealing in air (D2 and D3) because the diamond is completely protected by the coating during the oxidation process.

To summarize, the boron carbide coating on the diamond particles was synthesized by heating the diamond particles in a powder mixture consisting of H_3_BO_3_, B and Mg in a vacuum. The amorphous content, bond state and coverage fraction of the boron carbide coating were strongly dependent on the synthesized temperature. The boron carbide coating prefers to grow on the diamond (100) surface rather than on the diamond (111) surface because atomic diffusion on the diamond (111) surface is more difficult. The diamond particle was completely covered by a stoichiometric B_4_C coating after holding the raw mixture at 1200 °C for 2 hours. The boron carbide coating on the diamond particles contributed to the enhancement of the oxidation resistance due to formation of a B_2_O_3_ oxygen barrier layer. In this study, all the boron carbide coatings were oxidized prior to the oxidation of diamond. Moreover, the B_2_O_3_ exhibits fluidity, which gives rise to secondary coating growth on the diamond particles (i.e., self-healing property), resulting in repair of defects (e.g., hole and blank). The coating on diamond can provide effective protection against oxidation by heating in air at 1000 °C for 1 h. In comparison to the uncoated diamond particles, the initial time prior to oxidation of diamond was delayed for 2 h. Furthermore, the boron carbide coating on the diamond particles also contributed to the maintenance of the static compressive strength during annealing in air.

## Method

Synthetic HPHT diamond particles (HSD90, particle size 70/80 mesh (180~212 μm), Henan huanghe whirlwind international Co., Ltd., China) were used. 20 g of the diamond particles were immersed in a mixture consisting of 10 g of boron (B), 5 g of magnesium (Mg) and 40 g of boric acid (H_3_BO_3_) powders. The diamond-powder mixture was mixed using vigorously mechanical stirring at room temperature for two hours. This mixture was placed on an alumina boat and placed into a tube furnace. The chamber was evacuated using a turbomolecular pump to 5×10^−3^ Pa prior to sample heating. The diamond-powder mixture was heated to 800, 1000 and 1200 °C for 2 hours to synthesize the boron carbide coating on the diamond particles. The vacuum was only broken when the furnace temperature reached room temperature. After cooling of the furnace, the samples were treated with dilute nitric acid to remove the soluble phases (including B_2_O_3_ and MgO) from the product. The coated diamonds were separated from the excess B powders using a sieve. The uncoated diamond particles are referred to as D0. In addition, the coated diamond particles synthesized at 800, 1000 and 1200 °C is referred to as D1, D2 and D3, respectively.

The microstructure of each sample was characterized by X-ray diffraction (XRD) using a Bruker D8 with a Cu Kα source. The chemical composition of the samples was determined using X-ray photoelectron spectroscopy (XPS) on a Physical Systems Quantum 2000 spectrometer with monochromatic Al Kα radiation. The samples used for XPS analysis were cleaned using Ar^+^ ion sputter etching with an energy of 1 keV to remove surface oxides. The compositions of the samples were determined from the XPS data using sensitivity factors calibrated from a boron carbide reference sample with a known composition. In all the measurements, the XPS analysis area was set to a diameter of 100 μm^43^, which was smaller than the diameter of the diamond particle (at least 180 μm). And the measurement area was selected using an *in-situ* X-ray beam induced secondary electron image. To obtain more information regarding the bonding conditions, the samples were also analysed by Raman spectroscopy using a Renishaw Micro Raman system 2000 with an excitation wavelength of 514 nm. The Raman analysis was performed on a confocal system to characterize the different crystal planes of the diamond particles. The surface morphologies and topographies of the films were characterized using a Hitachi S-4800 scanning electron microscope (SEM). All the samples were annealed at 1000 °C with a heating rate of 5 °C min^–1^ in an air atmosphere to investigate the oxidation resistance. After annealing, the uncoated diamond particles (D0) are referred to as A0. After annealing, the corresponding samples of D1, D2 and D3 are referred to as A1, A2 and A3, respectively. Thermal gravimetric analysis (TGA) was performed using a Netzsch STA449F3. The temperature of the TGA was increased from room temperature (20 °C) to 1000 °C at a rate of 5 °C/min, and then, the temperature was maintained at 1000 °C for 4 h. An air atmosphere was flowed through the chamber during the measurement. The static compressive strength of one diamond particle was measured by continuously adding load until the particle broken. At least forty particles were measured for each sample to obtain higher measurement accuracy.

## Additional Information

**How to cite this article**: Sun, Y. *et al.* Enhancement of oxidation resistance via a self-healing boron carbide coating on diamond particles. *Sci. Rep.* **6**, 20198; doi: 10.1038/srep20198 (2016).

## Figures and Tables

**Figure 1:** XRD spectra for uncoated diamond particle (D0) and diamond particles with a boron carbide coating synthesized at 800 (D1), 1000 (D2) and 1200 °C (D3).

**Figure 2:** XPS (**a**) C1s and (**b**) B1s spectra for the boron carbide coatings on the diamond (100) surface that were synthesized at 800 (D1), 1000 (D2) and 1200 °C (D3).

**Figure 3:** Raman spectra of the uncoated diamond (100) surface (D0) and boron carbide coating on the diamond (100) surface synthesized at 800 (D1), 1000 (D2) and 1200 °C (D3).

**Figure 4:** SEM images for (**a**) typical uncoated diamond particles (D0) and diamond particles with coating synthesized at (**b**) 800 (D1), (**c**) 1000 (D2) and (**d**) 1200 °C (D3). The inset images in (**b**) and (**c**) show details of the coating on the diamond (111) surface with an enlarged scale.

**Figure 5:** Typical SEM cross-section image for the boron carbide coating on the diamond (**a**) (100) and (**b**) (111) surfaces synthesized at 1200 °C (D3).

**Figure 6:** XRD spectra of the uncoated diamond particles (A0) and diamond particles with boron carbide coating synthesized at 800 (A1), 1000 (A2) and 1200 °C (A3) after annealing in air.

**Figure 7:** XPS (**a**) B1s and (**b**) O1s spectra of the boron carbide coating on the diamond (100) surface synthesized at 800 (A1), 1000 (A2) and 1200 °C (A3) after annealing in an air atmosphere.

**Figure 8:** Raman spectra of the uncoated diamond surface (A0) and boron carbide coating on the diamond (100) surface synthesized at 800 (A1), 1000 (A2) and 1200 °C (A3) after annealing.

**Figure 9:** TGA results for the uncoated diamond particles (D0) and diamond particles with boron carbide coating synthesized at 800 (D1), 1000 (D2) and 1200 °C (D3). Drawing of partial enlargement is provided to show the weight gain in detail.

**Figure 10:** SEM images of the (**a**) typical uncoated diamond particles (A0) and diamond particles with boron carbide coating synthesized at (**b**) 800 (A1), (**c**) 1000 (A2) and (**d**) 1200 °C (A3) after annealing.

**Figure 11:** Static compressive strengths for the uncoated diamond particles (D0) and diamond particles with the boron carbide coating synthesized at 800 (D1), 1000 (D2) and 1200 °C (D3), and the results for the corresponding samples (A0-3) after annealing.

**Figure 12:** Relationship between the initial temperature of the weight gain observed in the TGA measurement and the amorphous content in the boron carbide coating on the diamond particles synthesized at different coating temperatures.

**Table 1:** Synthesis temperature, composition, B:C atomic ratio, bond fraction and amorphous content for the boron carbide coatings on the diamond (100) surface synthesized at 800 (D1), 1000 (D2) and 1200 °C (D3).

NO.	T (°C)	Composition (at.%)		B:C	Bond Fraction in C1s (%)		Bond Fraction in B1s (%)		Amorphous content (%)
		C	B		C-C	C-B	B-C*	B-C	
D1	800	25	75	3:1	25	75	30	70	29
D2	1000	22	78	3.6:1	13	87	14	86	14
D3	1200	20	80	4:1	3	97	0	100	1

**Table 2:** Composition and B:O ratio for the coatings on the diamond (100) surface after annealing as well as the parameters for the annealing process.

NO.	Annealing Temperature (°C)	Heating Rate (°C/min)	Composition			B:O
			C (at.%)	B (at.%)	O (at.%)	
A1	1000	5	6	38	56	2:3
A2	1000	5	3	39	58	2:3
A3	1000	5	1	40	59	2:3
